# Application Value and Relevance Analysis of the Risk Evaluation System for Arteriovenous Fistula Puncture in Thrombosis after Puncture

**DOI:** 10.1155/2021/6919979

**Published:** 2021-12-02

**Authors:** Mei Li, Chao Sun, Xuan Du

**Affiliations:** ^1^Department of Blood Purification Center, Qingdao Municipal Hospital, Qingdao 266011, Shandong, China; ^2^Department of High Pressure Oxygen Family, Qingdao Municipal Hospital, Qingdao 266011, Shandong, China; ^3^Department of Hepatobiliary Surgery, Qingdao Municipal Hospital, Qingdao 266011, Shandong, China

## Abstract

**Objective:**

To analyze the application value and relevance of risk evaluation system for arteriovenous fistula (AVF) puncture in thrombosis after puncture.

**Methods:**

The clinical data of 180 patients treated with hemodialysis in the hemodialysis center of our hospital from November 2017 to November 2019 were retrospectively analyzed. After puncture, all patients received the digital subtraction angiography (DSA) examination, and based on whether they had AVF thrombosis, they were divided into the nonthrombosis group (*n* = 102) and thrombosis group (*n* = 78), and then, according to the parity of their admission numbers, the patients in the thrombosis group were subdivided into the study group (*n* = 39) and the reference group (*n* = 39), so as to analyze the risk factors of thrombosis after AVF puncture and the application value of the risk evaluation system for AVF puncture in preventing and treating thrombosis.

**Results:**

Compared with the reference group after intervention, the study group had significantly higher mean internal fistula blood flow volume (*P* < 0.001) and significantly lower total incidence rate of vascular complications in fistulas (*P* < 0.05); according to the multifactor binary logistic regression analysis, it was found that diabetes, systolic blood pressure reduction, hemoglobin, low-density lipoprotein cholesterol (LDL-C), ultrafiltration rate, and elevation of blood phosphorus and platelet levels were the risk factors of thrombosis after AVF puncture in hemodialysis patients.

**Conclusion:**

When risk factors of thrombosis are found in patients treated with hemodialysis, timely detection and intervention shall be applied in the early stage. Adopting the AVF puncture risk evaluation system has an extremely high application value in the clinic and is of important meaning in prolonging the service life of fistulas.

## 1. Introduction

Kidney disease has become an important disease that endangers human life health [1]. Investigations have found that at least 2.4 million people die each year from kidney disease, which is currently the 11^th^ leading cause of global mortality [2, 3]. Hemodialysis therapy is a common technique in the treatment of kidney disease, which can replace the kidney to complete metabolic function in order to prolong survival [4]. Arteriovenous fistulas (AVFs) are the more important vascular access in hemodialysis, which have longer life and can ensure the smooth implementation of hemodialysis treatment and reduce the impact on the normal life of patients [5]. However, the inappropriate puncture method and higher puncture failure rate during dialysis will increase the damage of internal fistula vessels in patients, leading to thrombosis and then causing the impairment of internal fistula function and threatening life [6, 7]. Interventional thrombolysis is a common method for treating thrombosis after puncture, which is based on the principle of combining thrombosis with drugs to achieve unobstructed blood flow through the dissolution process. However, this treatment may trigger complications such as local or even organ hemorrhage. The AVF puncture risk evaluation system is a clinical risk evaluation method summarized and developed by reviewing the previous literature and interviewing the hemodialysis specialist nurses. Through the analysis of the current risk factors of patients undergoing dialysis, a systematic and standardized puncture evaluation system is provided for patients to reduce thrombosis, enhance the success rate of AVF puncture, and prolong their survival [8, 9]. The application value of AVF puncture risk evaluation system in thrombosis after puncture and their relevance were analyzed in the study, with the results summarized as follows.

## 2. Data and Methods

### 2.1. General Information

The clinical data of 180 patients treated with hemodialysis in the hemodialysis center of our hospital from November 2017 to November 2019 were retrospectively analyzed. Based on whether they had AVF thrombosis after puncture, they were divided into the nonthrombosis group (*n* = 102) and thrombosis group (*n* = 78), and then, according to the parity of their admission numbers, the patients in the thrombosis group were subdivided into the study group (*n* = 39) and the reference group (*n* = 39).

### 2.2. Inclusion and Exclusion Criteria

Inclusion criteria were as follows: AVFs were used as the treatment access during hemodialysis, the condition was not seriously progressed, the patients had good cognition and compliance, and the study met the World Medical Association Declaration of Helsinki (2013) [10].

Exclusion criteria were as follows: patients with less than 3 months of usage of AVFs for puncture after AVFs were mature, patients with acute active hemorrhagic disease, and patients with cachexia or severe malnutrition.

### 2.3. Methods

Clinical intervention was performed to patients with thrombosis after puncture of AVFs. Postoperative clinical routine intervention was conducted to the patients in the reference group, including easing their negative emotions, encouraging them to keep a good mood, and carrying out health education around the principles of dialysis, precautions for fistula nursing, and personal hygiene, supplementing blood volume, correcting low blood pressure, implementing thrombolytic therapy when necessary, and pressing the injection part with moderate stress at the end of thrombolytic therapy every time to avoid vascular embolism in fistula again [11, 12].

The risk evaluation system for puncture of AVFs was carried out in the study group with the following specific steps. A risk evaluation group was established, including 1 professor from the nephrology department, 1 physician from the hemodialysis center, and 3 specialist nurses, and by means of reviewing relevant literature and interview, an initial evaluation index item pool was built, and an expert consultation questionnaire was compiled to count and analyze the relevant data after distribution and collection. Based on the principles of index screening and by combining with the suggestions and opinions proposed by the experts, the group members revised the initial indexes, deleted gender and BMI values and 5 corresponding evaluation criteria, added the history of intubation at the fistula side, fistula blood flow volume, degree of vessel exposure, times of fistula establishment, and corresponding evaluation criteria, modified peripheral arterial disease into vasculopathy, fistula tremor, and murmur into fistula tremor and fistula murmur, and fistula service time into fistula service life, thus finally forming the evaluation index system for risk factors of AVF puncture, which included 4 first-level indexes, 21 second-level indexes, and 52 evaluation criteria for the second-level indexes.

### 2.4. Study Methods

The clinical data of 180 patients who accepted hemodialysis in the hemodialysis center of our hospital were collected, including their age, gender, dialysis duration, diastolic blood pressure, and systolic blood pressure, and relevant laboratory indexes were measured, including platelet, triacylglycerol (TAG), hemoglobin, and blood phosphorus. The patients' fistula blood flow volume was measured with the color doppler ultrasonic diagnostic apparatus (manufactured: Shanghai Mingyuan Industry Company Ltd.; model: DW-T8) by the same doctor from the ultrasonographic department. One cm from the vein side at fistula anastomotic stoma was checked, the fistula orifice was exposed to measure the caliber, the color doppler was overlaid to show the blood flow direction and obtain the blood flow spectrum of fistula, the spectrum area was drawn with the vernier to obtain the practical integral velocity *V*_min_, the fistula blood volume was calculated according to the formula AVFB = *π*D^2^/(4 × 60 × *V*_min_) [13], and the occurrence of vascular complications of fistula after intervention of the two groups was counted.

### 2.5. Statistical Methods

Table 1 provides the details of statistical methods used.

## 3. Results

### 3.1. Comparison of Patients' Baseline Information between the Thrombosis Group and Nonthrombosis Group

The systolic blood pressure, hemoglobin, number of patients with combined diabetes, low-density lipoprotein cholesterol (LDL-C), ultrafiltration rate, blood phosphorus, and platelet levels in patients of the two groups were significantly different (*P* < 0.05), and other indicators presented no significant difference (*P* > 0.05), as given in Table 2.

### 3.2. Comparison of Fistula Blood Flow Volume after Intervention between the Two Groups

After intervention, the mean fistula blood flow volume of the study group was significantly higher than that of the reference group (*P* < 0.001), as shown in Figure 1.

### 3.3. Comparison of Incidence Rates of Fistula Vascular Complications after Intervention between the Two Groups

After intervention, the total incidence rate of fistula vascular complications was significantly lower in the study group than in the reference group (*P* < 0.05), as given in Table 3.

### 3.4. Multifactor Analysis on Thrombosis after AVF Puncture in Patients Undergoing Hemodialysis

Taking the thrombosis group (1) and nonthrombosis group (2) as the dependent variables and the factors indicating *P* < 0.05 in single-factor analysis as the independent variables to carry out multifactor binary logistic analysis, it was found that diabetes, systolic blood pressure reduction, hemoglobin, LDL-C, ultrafiltration rate, blood phosphorus, and elevation level of platelet were considered as the risk factors for thrombosis after AVF puncture in patients undergoing hemodialysis (Table 4).

### 3.5. Relevance of Thrombosis after AVF Puncture

Figure 2 shows the relevance of thrombosis after AVF puncture.

### 3.6. Comparison of Areas, SE^a^, Asymp.sig.^b^, and Asymp. 95% CI among Various Indexes

Table 5 provides the comparison of area, SE^a^, Asymp.sig.^b^, and Asymp. 95% CI among various indexes.

### 3.7. Comparison of Positive Rates, Sensitivity, and Specificity among Various Indexes

Platelet presented the highest sensitivity, while LDL-C had the highest specificity, as given in Table 6.

## 4. Discussion

Epidemiological studies have shown that [14] the incidence rate of renal disease in China is about 13%, hemodialysis is the common method to treat renal failure, and effective and well-functioning vascular access is the fundamental guarantee to perform long-term sustained hemodialysis [15–17]. Currently, AVF puncture has become the first choice to establish vascular access in the clinic because of fewer complications, high patency rate, and low cost [18]. However, with the influence of long-term use and various factors, the internal fistula will gradually narrow and harden, leading to thrombosis, decrease of function, and life shortening, and seriously endangering the life of patients [19]. Therefore, actively searching for efficient clinical management measures is of great significance to reduce thrombosis after AVF puncture.

The risk evaluation system for AVF puncture can help patients in maintaining good vascular access and is essential to improve the quality of survival and reduce the cost of diagnosis and treatment for dialysis patients [20]. In this study, the routine clinical nursing intervention and risk evaluation system were, respectively, implemented to patients with thrombosis after AVF puncture, and the experimental results showed that the mean fistula blood flow volume after intervention was significantly higher in the study group than in the reference group (*P* < 0.001), indicating that the risk evaluation system could effectively improve the blood flow of autologous AVFs in hemodialysis patients, had a certain effect on preventing the formation of scar on the skin and surrounding of fistula, and obtained a good clinical effect.

Thrombosis after puncture is an important reason affecting the therapeutic effect of dialysis in patients [21]. In this study, by exploring the risk factors of thrombosis in AVFs of hemodialysis patients and carrying out multifactor binary logistic analysis, it was concluded that diabetes, systolic blood pressure reduction, hemoglobin, LDL-C, ultrafiltration rate, elevation of blood phosphorus, and platelet were the risk factors for thrombosis after AVF puncture in hemodialysis patients. It has been found that the proportion of thrombosis, whether it is initial or relapsed, is high in patients with diabetes mellitus because such disease can participate in the formation of internal fistula thrombosis by means of causing human vascular endothelial injury and vascular atherosclerosis [22, 23] to be specific, poor long-term glycemic control, and increased glycosylation end products cause elevated levels of related inflammatory factors and then injure the tunica intima, which, combined with the disturbed lipid metabolism in the body, contribute to the progression of atherosclerosis and can also lead to the formation of fistula thrombosis [24]. It is a viewpoint that had been confirmed in the study by He Qing et al. [25], suggesting that AVF thrombosis is related to the hypercoagulable state in patients. The ROC curves of the indexes showed that the area under the platelet curve was the largest, which is due to the close relationship between the platelet function changes and the incidence of thrombosis. The changes of blood vessels, blood flow, and blood components can lead to thrombosis, and platelet undergoes aggregation, adhesion, and secretion reactions while participating in thrombosis, thus resulting in vascular endothelial injury. Therefore, the measurement of platelet after puncture can play a role in preventing and reducing thrombosis. By calculating the positive rates, sensitivity, and specificity of the indexes, it was found that LDL-C had the highest positive rate. In clinical research, negative and positive are ways to judge the experimental results, and the positive results are of great significance to doctors and patients, which can further illustrate that the risk of thrombosis can be judged after measuring the LDL-C level of patients after puncture. Further analysis in this study showed that platelet presented the highest sensitivity, while LDL-C had the highest specificity. Higher diagnostic sensitivity suggests higher diagnostic accuracy of this index for this disease. The specificity, also known as the true negative rate, reflects the ability of screening tests to determine nonpatients. Therefore, the measurement of above indexes in hemodialysis patients should be strengthened in the clinic, and targeted prevention and nursing measures should be adopted to reduce the occurrence of fistula thrombosis as much as possible. Deficiencies of the study are as follows: the cases selected herein were the patients treated in our hospital; hence, the source of cases lacked diversity; in addition, because the influence of factors such as patients' age and blood pressure on fistula thrombosis was less and might be covered by other factors, and deviation of study results may appear. To sum up, the initial conclusion obtained by the study shall be perfected by future research.

## 5. Conclusion

In conclusion, when risk factors of thrombosis are found in patients treated with hemodialysis, timely detection and intervention shall be applied in the early stage. Adopting the AVF puncture risk evaluation system has extremely high application value in the clinic and is of important meaning in prolonging the service life of fistulas.

## Figures and Tables

**Figure 1:** Comparison of fistula blood flow volume after intervention between the two groups (mean ± SD). The horizontal axis indicates the study group and the reference group, and the vertical axis indicates the fistula blood volume in ml/min. After intervention, the mean fistula blood flow volume of the study group and the reference group was 734.50 ± 21.72 and 560.97 ± 45.42, respectively.  ^*∗*^Significant difference in the mean fistula blood flow volume after intervention between the two groups (*t* = 31.117, *P* < 0.001).

**Figure 2:** Relevance of thrombosis after AVF puncture.

**Table 1:** 

Methods	Application
SPSS 23.0	Data processing and ROC curve drawing
GraphPad Prism 7	Picture drawing
Logistic retrospective analysis	Related risk factors analysis

**Table 2:** Comparison of baseline information between the thrombosis group and nonthrombosis group.

Item	Thrombosis group (*n* = 78)	Nonthrombosis group (*n* = 102)	*X* ^2^/*t*	*P*
Gender			0.063	0.802
Male/female	42/36	53/49		
Mean age (mean ± SD, years)	57.26 ± 2.36	57.31 ± 2.32	0.142	0.887
BMI (mean ± SD, kg/m^2^)	21.16 ± 1.26	21.21 ± 1.19	0.272	0.786
Systolic blood pressure (mmHg)	126.24 ± 9.62	132.36 ± 8.82	4.435	<0.01
Dialysis duration (months)	16.27 ± 2.36	16.35 ± 2.25	0.231	0.817
Diastolic blood pressure (mmHg)	82.36 ± 6.47	81.83 ± 6.54	0.541	0.589
Hemoglobin (g/L)	103.27 ± 7.28	93.16 ± 7.16	9.320	<0.01
TAG (mmol/L)	1.73 ± 0.69	1.85 ± 0.71	1.137	0.257
Total cholesterol (mmol/L)	5.24 ± 2.16	4.63 ± 2.06	1.928	0.056
LDL-C (mmol/L)	3.02 ± 0.46	2.51 ± 0.61	6.163	<0.01
HDL-C (mmol/L)	1.31 ± 0.36	1.37 ± 0.28	1.258	0.210
Ultrafiltration rate (ml/min)	10.36 ± 2.43	6.26 ± 2.16	11.951	<0.01
Diabetes	20 (25.64)	41 (40.20)	4.179	0.041
Serum phosphorus (mmol/L)	2.14 ± 0.36	1.59 ± 0.29	11.350	<0.01
Hemoglobin (g/L)	81.26 ± 1.27	77.32 ± 1.34	19.993	<0.01
Platelet (×109/L)	218.26 ± 15.28	179.21 ± 15.34	16.953	<0.01

Smoking history				
Yes/no	24/54	39/63	1.083	0.298

Drinking history				
Yes/no	31/47	51/51	1.875	0.171

Marital status				
Married	71 (91.03)	90 (88.24)	0.365	0.546
Unmarried	5 (6.41)	7 (6.86)	0.015	0.904
Divorced	2 (2.56)	5 (4.90)	0.646	0.421

Educational degree				
College	4 (5.13)	9 (8.82)	0.901	0.343
Secondary school	34 (43.59)	48 (47.06)	0.215	0.643
Primary school	40 (51.28)	46 (45.10)	0.678	0.410

Place of residence			0.479	0.489
Urban area	40 (51.28)	47 (46.08)		
Rural area	38 (48.72)	55 (53.92)		

**Table 3:** Comparison of incidence rates of fistula vascular complications after intervention between the two groups (*n* (%)).

Group	*n*	False aneurysm	Acute cardiac insufficiency	Arteriovenous anastomotic rupture bleeding	Graft infection	Total incidence rate
Study	39	0 (0.00)	1 (2.56)	1 (2.56)	0 (0.00)	5.13% (2/39)
Reference	39	3 (7.69)	2 (5.13)	2 (5.13)	1 (2.56)	20.51% (8/39)
*X* ^2^						4.129
*P*						＜0.05

**Table 4:** Analysis of relevant factors for thrombosis after AVF puncture.

Item	HR	95% CI	*P*
Systolic blood pressure	1.273	0.936–1.626	0.017
Diastolic blood pressure	1.036	0.527–1.417	0.835
Dialysis duration	1.736	1.352–2.142	0.362
Systolic blood pressure	0.634	0.418–1.215	<0.001
TAG	0.927	0.682–1.136	0.825
LDL-C	1.835	1.146–2.317	0.024
Hemoglobin	1.036	0.728–1.216	0.004
HDL-C	0.936	0.638–1.243	0.528
Ultrafiltration rate	1.015	0.758–1.326	0.021
Blood phosphorus	1.638	1.063–2.231	0.003
Diabetes	1.274	0.862–1.628	0.031
Platelet	0.618	0.528–1.246	0.026

**Table 5:** Area under curve.

Variable of test results	Area	SE^a^	Asymp.sig.^*b*^	Asymp. 95% CI	
				Lower limit	Upper limit
Systolic blood pressure	0.850	0.032	0.000	0.788	0.912
Platelet	0.937	0.021	0.000	0.895	0.979
Diabetes	0.887	0.028	0.000	0.832	0.941
LDL-C	0.909	0.025	0.000	0.861	0.957
Ultrafiltration rate	0.902	0.026	0.000	0.850	0.953
Blood phosphorus	0.867	0.029	0.000	0.810	0.924
Hemoglobin	0.887	0.028	0.000	0.832	0.941

**Table 6:** Diagnosis results of various indexes.

Index	Systolic blood pressure	Platelet	Diabetes	LDL-C	Ultrafiltration rate	Blood phosphorus	Hemoglobin
Positive (cases)	63	72	68	73	68	71	68
Positive rate (%)	35.00	40.00	37.78	40.56	37.78	39.44	37.78
Sensitivity (%)	87.64	93.98	88.64	86.67	91.76	81.25	88.64
Specificity (%)	87.18	94.44	91.07	95.33	91.07	93.58	91.07

## Data Availability

The data used to support the findings of this study are available from the corresponding author upon request.
